The article "Nonocclusive Mesenteric Ischemia Associated with Ogilvie Syndrome" was published in 2014. Journal: Case Rep Surg.

# Nonocclusive Mesenteric Ischemia Associated with Ogilvie Syndrome

**DOI:** 10.1155/2014/821832

**Published:** 2014-09-07

**Authors:** Takashi Sakamoto, Toshiyuki Suganuma, Shinichiro Okada, Kensuke Nakatani, Sawako Tamaki, Alan T. Lefor

**Affiliations:** ^1^Department of Surgery, Tokyo Bay Urayasu Ichikawa Medical Center, 3-4-32 Todaijima, Urayasu, Chiba, Japan; ^2^Department of Surgery, Yokosuka General Hospital Uwamachi, Kanagawa, Japan; ^3^Department of Surgery, Jichi Medical University, Tochigi, Japan

## Abstract

Nonocclusive mesenteric ischemia (NOMI) is one type of acute mesenteric ischemia. Colonic pseudoobstruction, known as Ogilvie syndrome, is a disorder defined by colonic distension in the absence of mechanical obstruction. A relationship between these diseases has not yet been reported, based on a review of the literature. We report a patient with NOMI secondary to Ogilvie syndrome. An 82-year-old woman reported three days of intermittent abdominal pain. Plain computed tomography scan showed colonic obstruction at the rectosigmoid colon. Colonoscopy was performed that showed a large amount of stool and no evidence of tumor or other physical causes of obstruction. We diagnosed the patient with Ogilvie syndrome and continued nonoperative management. On the third hospital day, she complained of abdominal distension. A repeat CT scan showed pneumatosis intestinalis in the small bowel and ascending colon, with portal venous gas. Emergency laparotomy was performed with diagnosis of mesenteric ischemia. Intraoperatively, there were multiple skip ischemic lesions in the small intestine and cecum. We resected the ischemic bowel and performed a distal jejunostomy. Her residual small bowel measured just 20 cm in length. Postoperatively, her general status gradually improved. She was discharged with total parenteral nutrition and a small amount of enteral nutrition.

## 1. Introduction

Nonocclusive mesenteric ischemia (NOMI) is one type of acute mesenteric ischemia, with diminished bowel perfusion which can result in intestinal necrosis, which is not due to a thrombus or embolus. The mortality of patients with NOMI is reported to be as high as 70 to 80% [1]. NOMI has been associated with a number of conditions including acute myocardial infarction with shock, congestive heart failure, arrhythmias, hypovolemia associated with pancreatitis, hemorrhage, sepsis, cirrhosis, and renal failure in patients undergoing dialysis [2]. Colonic pseudoobstruction, known as Ogilvie syndrome, is a disorder defined by colonic distension in the absence of mechanical obstruction, and the pathogenesis is not well known. Ogilvie syndrome sometimes requires laparotomy to establish the diagnosis but in general has a good prognosis, usually without the need for surgical intervention.

A relationship between these two diseases has not yet been reported, based on a review of the literature. We report a patient with NOMI which we believe may be secondary to Ogilvie syndrome.

## 2. Case Report

An 82-year-old woman with a history of hypertension, lipid disturbance, chronic constipation, and insomnia reported three days of intermittent abdominal pain and vomiting, which prompted ambulance transport to the emergency department. She had a slightly impaired performance status. The pain began gradually in the right lower abdomen and became generalized in the abdomen on the day before admission, accompanied by an episode of vomiting.

On admission, the patient's vital signs were normal. Physical examination showed that her oral cavity was dry and her abdomen was soft and distended, with hyperactive bowel sound and tenderness in the right lower quadrant. There were no peritoneal signs on physical examination. Rectal examination showed normal sphincter tone and no apparent tumor. Laboratory tests revealed an elevated white blood cell count, blood urine nitrogen, and creatinine, at 9400/*μ*, 50.9 mg/dL, and 1.07 mg/dL, respectively. Plain computed tomography scan showed colonic obstruction at the rectosigmoid colon (Figure 1). The colon was filled with stool proximally and the cecum measured 95 mm.

Based on these findings, we suspected colonic pseudoobstruction, Ogilvie syndrome, partly because she had undergone a negative colonoscopy one year previously. We stopped her medications including calcium channel blocker and benzodiazepine, which can affect bowel motility. On the second hospital day, colonoscopy was performed for diagnosis and treatment that showed a large amount of stool and no evidence of tumor or other physical causes of obstruction. Her abdominal pain and distension were relieved after the procedure. We diagnosed the patient with Ogilvie syndrome and continued to withhold oral intake providing her with parenteral nutrition and began subcutaneous neostigmine. After endoscopic reduction, watery diarrhea was seen.

On the third hospital day, the diarrhea stopped, her blood pressure decreased, and she developed oliguria. Her blood pressure did not respond to crystalloid infusion, and she complained of abdominal distension with mild pain. Physical examination showed diffuse tenderness throughout the abdomen without peritoneal signs. We suspected obstruction and a repeat CT scan showed massive pneumatosis intestinalis in the small bowel and ascending colon, with superior mesenteric venous gas and hepatic portal venous gas (Figures 2(a) and 2(b)). Serum lactate level was 6.7 mmol/L, and she was diagnosed with mesenteric ischemia.

Emergency laparotomy was immediately performed. Intraoperatively, there were multiple skip ischemic lesions in the small intestine and cecum (Figure 3). Pulsation was palpable in the superior mesenteric artery, but not in the ileocecal and middle colonic arteries. Based on these findings, we decided to resect the ischemic bowel and performed a distal jejunostomy. Her residual small bowel measured just 20 cm in length. Pathological examination of the resected intestine showed air in the vessels and no thrombosis in the mesenteric marginal artery. Only a few centimeters of proximal and distal intestine were not necrotic, but there were many patchy necrotic lesions in the specimen.

Postoperatively, she was brought to the intensive care unit with continued mechanical ventilation. Her general status and vital signs gradually improved. On the third postoperative day, she was extubated and she was transferred to a regular ward. The output from the jejunostomy did not change from about 1200 mL/day throughout the postoperative period. We started total parenteral nutrition on postoperative day 11 and a small amount of enteral nutrition on postoperative day 37. She was discharged on postoperative day 41 with total parenteral nutrition, little enteral nutrition, and the same performance status as on admission.

## 3. Discussion

Colonic pseudoobstruction, also known as Ogilvie syndrome, is a disorder defined as colonic distension in the absence of mechanical obstruction, which was first described in 1948 by Sir William Heneage Ogilvie [3]. The mechanism of colonic pseudoobstruction is not understood. The diagnosis is made based on the clinical presentation and radiological studies. Clinical findings include abdominal distension, abdominal pain, and nausea or vomiting. In patients with severe abdominal pain or fever, perforation with or without ischemia should be considered. In the present patient, she had mild tenderness and abdominal distension, with mild leukocytosis on arrival, but there were no definite peritoneal signs on physical examination and she was afebrile. Initial imaging studies showed no free air.

The rate of perforation in this condition is reported to be about 3% [4] and is generally associated with a cecal diameter greater than 12 cm [5]. The strategy for the management of patients with colonic pseudoobstruction depends on the presence of perforation or ischemia. Nonoperative management including bowel rest, administration of intravenous fluids, and correction of electrolyte abnormalities is recommended in patients without perforation or ischemia. The reported success of nonoperative management is variable, with rates reported from 20% to 92% [6]. Colonoscopic decompression is recommended in patients who do not respond to nonoperative management within 24 hours. This approach has been reported to be successful in approximately 80% of patients, but up to 20% will require repeat endoscopy due to recurrence [7]. If perforation occurs, the mortality rate is as high as 50% [8], and surgical management is mandatory.

Generally, acute mesenteric ischemia is classified into subtypes depending on the etiology, including superior mesenteric artery embolus, NOMI, superior mesenteric artery thrombosis, and acute mesenteric venous thrombosis. NOMI is not caused by a dominant thrombus or embolus but is rather caused by a low flow state, with the highest mortality among all causes of acute mesenteric ischemia. The mortality rate of patients with NOMI is reported to be as high as 70 to 80% [1].

NOMI has been associated with a wide range of conditions, such as patients who underwent cardiopulmonary bypass or are undergoing hemodialysis [9]. Drugs such as cocaine, epinephrine, norepinephrine, vasopressin, and digoxin may cause splanchnic vasoconstriction resulting in NOMI [10, 11]. While the majority of patients with acute mesenteric ischemia have abdominal pain, some patients with NOMI do not experience pain presenting only with abdominal distension [3]. Patients with NOMI benefit from early diagnosis but establishing the diagnosis may be difficult. Plain X-rays, duplex sonography, computed tomography, and magnetic resonance imaging have limited value. Angiography is still the only test to definitively establish the diagnosis of NOMI [10].

There is controversy about using angiography in patients with acute abdominal findings, because the presence of peritoneal signs may be an indication of infarcted bowel needing laparotomy. It is difficult to perform angiography in such a critically ill patient. In this patient, computed tomography scan showed pneumatosis intestinalis and portal vein gas, indicating bowel necrosis [12]. Pneumatosis intestinalis with portomesenteric venous gas correlates strongly with transmural bowel infarction [12]. Therefore, it was appropriate to proceed with immediate laparotomy without first obtaining visceral angiography in this patient because there was little doubt about the diagnosis. In some situations early angiography is useful and can determine the cause, that is, embolic ischemia versus NOMI, providing a “roadmap” for the surgeon at laparotomy.

Ischemia in patients with pseudoobstruction is well known, but previous reports have described colonic ischemia [5]. NOMI of the superior mesenteric artery after colonic pseudoobstruction has not been previously reported. In this patient, one hypothesis is that pseudoobstruction with hypovolemia due to watery diarrhea after endoscopic decompression might have led to the development of NOMI. A large amount of crystalloid was administered after endoscopic decompression. Her past medical history did not include heart disease or renal failure. Neostigmine administration is one of the supportive measures but is contraindicated in a patient with perforation and ischemia. We also hypothesize that neostigmine may have led to ischemia by increasing the motility of the small bowel leading to increased oxygen demand. It is difficult to determine the pathogenesis of NOMI in this patient. This suggests the careful administration of neostigmine in the elderly with Ogilvie syndrome.

## 4. Conclusion

NOMI is a relatively rare cause of abdominal pain but patients have significant mortality. Patients with Ogilvie syndrome have a relatively good prognosis. Acute mesenteric ischemia from a variety of causes, including NOMI, needs a prompt diagnosis and urgent management to limit mortality. It is difficult to suspect NOMI in patients who already have a diagnosis to explain their abdominal pain. NOMI is associated with many conditions that result in hypovolemia. NOMI must be considered in the differential diagnosis, even in patients with an established diagnosis to explain their abdominal pain.

## Figures and Tables

**Figure 1:** Plain computed tomography scan shows a dilated cecum measuring 95 mm.

**Figure 2:** (a) Pneumatosis intestinalis is seen in the small bowel and ascending colon. (b) Portal vein gas is present in the liver.

**Figure 3:** Multiple skip ischemic lesions in the small intestine are seen at laparotomy.

## References

[1] Schoots IG, Koffeman GI, Legemate DA, Levi M, van Gulik TM (2004). Systematic review of survival after acute mesenteric ischaemia according to disease aetiology. *British Journal of Surgery*.

[2] Michael JS (2014). Acute mesenteric ischemia. *Surgical Clinics of North America*.

[3] Kozuch PL, Brandt LJ (2005). Review article: diagnosis and management of mesenteric ischaemia with an emphasis on pharmacotherapy. *Alimentary Pharmacology & Therapeutics*.

[4] Rex DK (1994). Acute colonic pseudo-obstruction (Ogilvie's syndrome). *The Gastroenterologist*.

[5] Vanek VW, Al-Salti M (1986). Acute pseudo-obstruction of the colon (Ogilvie's syndrome). An analysis of 400 cases. *Diseases of the Colon and Rectum*.

[6] Harrison ME, Anderson MA, Appalaneni V (2010). The role of endoscopy in the management of patients with known and suspected colonic obstruction and pseudo-obstruction. *Gastrointestinal Endoscopy*.

[7] de Giorgio R, Knowles CH (2009). Acute colonic pseudo-obstruction. *British Journal of Surgery*.

[8] Saunders MD (2007). Acute colonic pseudo-obstruction. *Best Practice and Research in Clinical Gastroenterology*.

[9] Brandt LJ, Boley SJ (2000). AGA technical review on intestinal ischemia. *Gastroenterology*.

[10] Bobadilla JL (2013). Mesenteric ischemia. *Surgical Clinics of North America*.

[11] Martin MC, Wyers MC (2014). Mesenteric vascular disease. *Rutherford's Vascular Surgery*.

[12] Gore RM, Yaghmai V, Thakrar KH (2008). Imaging in intestinal ischemic disorders. *Radiologic Clinics of North America*.

